# Lateral Circumflex Femoral Vascular Chimeric Fascia Flap Reduces Pain and Promotes Wound Healing in Repairing Skin and Tendon Defects of Hand, Foot, and Ankle

**DOI:** 10.1155/2022/2874332

**Published:** 2022-07-30

**Authors:** Liming Xu, Jianshun Zhang, Faliang Shi, Renkuan Wang, Jianyan Wu

**Affiliations:** ^1^Microsurgery, Jiaozhou Branch of Shanghai East Hospital, Tongji University, Jiaozhou, China; ^2^Functional Division, Jiaozhou Branch of Shanghai East Hospital, Tongji University, Jiaozhou, China; ^3^Joint Surgery, Qingdao West Coast New District People's Hospital, Qingdao, China; ^4^Department of Anesthesiology, Jiaozhou Branch of Shanghai East Hospital, Tongji University, Jiaozhou, China

## Abstract

The purpose of this study was to investigate the clinical efficacy of lateral circumflex femoral artery embedded with fascia lata flap in the repair of skin and tendon defects in hand, foot, and ankle. From January 2020 to June 2021, 32 patients with skin and tendon defects of the hand, foot, and ankle admitted to our hospital were selected as the study subjects. According to the random number table method, they were divided into the observation group (16 cases, treated with rotational lateral femoral vascular inlay broad fascial flap repair) and the control group (16 cases, treated with conventional skin flap repair) and followed up for 6 months. The postoperative tendon midactivity measurement scale (TAM), ankle-hindfoot scoring system (AOFAS), and lower limb functional evaluation scale (LEFS) scores were all higher in the observer group than in the control group The number of people with infection, implant necrosis, and subcutaneous hematoma in the observation group (total incidence 6.25%) was less (lower) than that in the control group (50.00%), and the total number of people with significant and fair clinical efficacy in the observation group (total effective rate 100.00%) was more (higher) than that in the control group (68.75%). The application of early plastic surgery to the clinical treatment of patients with deep burns on the hand can reduce the patient's pain and promote the healing of the wound. It is of great significance to reduce the risk of complications such as necrosis of the skin graft and improve the efficacy of the surgery.

## 1. Introduction

Cutaneous defects of the hand, foot, and ankle are tissue defects that involve the skin. Depending on the severity of the defect, it can be divided into simple defects (superficial skin and soft tissue only) and complex defects (deep muscle, tendon, and bone defects in addition to skin), i.e., skin and tendon defects of the hand, foot, and ankle are the more serious complex defects [1, 2]. It is typically characterized by localized pain and impaired movement and, if not treated promptly, can cause serious impairment to the function of the affected limb, resulting in a reduced quality of life [3, 4]. In clinical practice, skin defects of the hand, foot, and ankle are mainly treated surgically, and conventional flap repair has limited effect and is not conducive to the recovery of motor function of the affected limb. The lateral femoral vascular inlay broad fascial flap repair not only provides an ideal flap donor area but also facilitates the repair of soft tissue and major vascular segments of the affected limb, which has a positive impact on the recovery of the motor function of the affected limb [5, 6]. In this study, 32 patients with skin and tendon defects in the hand, foot, and ankle admitted to our hospital from January 2020 to June 2021 were compared between conventional skin flap repair and rotated lateral femoral vascular inlay broad fascial flap repair treatment. It further provides a reference for the clinical diagnosis and treatment of skin and tendon defects in hands, feet, and ankles.

## 2. Patients and Methods

### 2.1. Patients

From January 2020 to June 2021, 32 patients with skin and tendon defects of the hand, foot, and ankle admitted to our hospital were selected as the study population. The inclusion criteria were as follows: (i) they met the criteria for treatment of skin and tendon defects of the hand, foot, and ankle [7]; (ii) they had typical symptoms such as swelling and pain and impaired movement; (iii) they had complete basic information; (iv) they were aged 18–65 years; (v) the patients and their families voluntarily signed the notification of information. Exclusion criteria were as follows: (i) patients with contraindications to surgery; (ii) patients with combined severe oncological disease; (iii) patients with severe coagulation dysfunction; (iv) patients with mental illness, language impairment, and low cooperation; (v) patients who withdrew from the study midway or those who were lost to follow-up. According to the random number table method, the patients were divided into the observation group (16 cases, treated with rotary lateral femoral vascular inlay broad fascial flap repair) and the control group (16 cases, treated with conventional skin flap repair). The differences were not statistically significant (*P* > 0.05) when comparing the basic data (age, area of skin lesion, length of tendon defect, and gender composition) of the two groups. See Table 1. The study was approved by the Jiaozhou Branch of Shanghai East Hospital Medical Ethics Committee.

### 2.2. Methods

Patients in the control group were treated as follows: conventional skin slice repair treatment. According to the patient's condition, a donor skin slice of appropriate size and shape (deep to the fat layer) is excised, full-thickness skin tissue was sharply excised, and full-thickness skin tissue for grafting was prepared in advance. After the patient was put under anesthesia, the necrotic tissue was removed from the wounded area, the shape and size of the recipient area were adjusted to match the donor skin slice, and the skin slice is grafted and sutured.

The patients in the observation group were treated as follows: the patients were treated with a rotated lateral femoral vascular inlay broad fasciocutaneous flap repair. (i) Flap and broad fascial preparation: ultrasound was used to locate and mark the superficial point of vascular skin penetration. Afterwards, the flap was marked along the donor flap, the entire flap and broad fascia are cut through the medial superior edge, the anterolateral femoral cutaneous nerve was cut, marked, and sutured to fix the broad fascia cutaneous edge and flap edge. The flap is turned out, the broad fascia and lateral femoral musculature were separated, the vascular tip of the main trunk of the lateral descending femoral branch (along the rectus femoris and lateral femoral muscle gap) was positioned, and the lateral branch of the descending branch is separated. The inner lower edge of the flap was incised, the vascular cutaneous branch was located and protected, the cutaneous branch (intramuscular) is freed retrogradely, the lateral femoral muscle was cut (partially), and the cutaneous branch of the lateral femoral muscle was separated by the “meeting method,” preserving 1-2 cutaneous branches to supply the flap. The skin was incised at the upper edge of the skin, and the anterior branch of the anterolateral femoral cutaneous nerve is marked around the patellar line and the flap was freed. An incision was made towards the distal thigh, and depending on the extent of the tendon defect in the affected limb, the corresponding length and width of about 4 cm of broad fascia were cut along the distal end of the flap, connecting the proximal end of the broad fascia to the distal end of the flap. (ii) Preparation of the recipient area: in the supine position, an epidural block was combined with a subarachnoid block. Once the patient was under anesthesia, the wound was cleared and rinsed with saline to locate the dorsalis pedis arteriosus, superficial peroneal nerve, or other cutaneous nerve branches in the recipient area. (iii) Graft repair treatment: the distal cut of the flap with the broad fascial myofascial surface turned out to form a cylinder is folded back and grafted to the tendon defect in the recipient area, the proximal severed end of the tendon is sutured (forming a bundle), the tendon line was sutured continuously, and then the distal and proximal ends were given appropriate tension according to the length of the tendon defect and treated with sutures. For extensor tendon defects of the thumb in the hand, the broad fascia can be cut longitudinally and divided into two bundles, with the radial bundle bridged to repair the thumb, with continuous sutures of the tendon cord, and the ulnar bundle sutured in the same way. For the vascular nerve anastomosis, microscopically anastomose the recipient artery and vein, the lateral branch artery and vein, and the lateral femoral cutaneous nerve and recipient cutaneous nerve with 9–0 sutures, respectively. The drainage tube was left in place, and the wound was sutured and closed.

Both groups received conventional anti-infection and anticoagulation treatment after surgery. Targeted rehabilitation exercises were given according to the patients' conditions. After discharge from the hospital, follow-up visits (6 months) were conducted by telephone and WeChat to provide postdischarge correction and guidance on diet and exercise rehabilitation and to advise the patients to be regularly re-examined in hospital.

### 2.3. Observation Indicators

The functional recovery of the affected limb was compared between the two groups: preoperatively and postoperatively (6 months after surgery), and the recovery of tendon, ankle, and lower limb function was assessed using the total activity measurement (TAM), the Ankle Hind foot Scale (AOFAS) and the Lower Extremity Functional Scale (LEFS). The TAM score was 3 for flexion of the finger end ≤3 cm from the palm, 2 for spacing <4 cm, 1 for spacing <5 cm, and 0 for spacing >5 cm or inability to flex the finger, with a positive correlation with tendon recovery; the AOFAS score includes pain (0–40 points), functional and voluntary activity support (0–10 points), maximum walking distance (0–5 points), ground walking (0–5 points), paradoxical walking (0–8 points), anterior-posterior activity (0–8 points), hind foot activity (0–6 points), ankle-hind foot stability (0–8 points), and foot alignment (0–10 points), a total of 0–100 points, with scores positively correlated with functional recovery of the foot and ankle. The LEFS scores totalled 20 subscales of 0–4 each, for a total of 0–80, and the scores were positively correlated with improvement in lower limb function.

Complications were compared between the two groups: the number of patients with infection, skin graft necrosis, and subcutaneous hematoma was counted.

The clinical outcomes of the two groups were compared: the recovery results achieved by the patients were counted from postoperative to 6 months of follow-up. Significant: TAM ≥2.50, AOFSA >74, good recovery of flap shape, color, and texture, close to the original skin, no complications such as necrosis of the implant; fair: 1.5 points ≤ TAM <2.5, 65 points < AOFSA ≤74, average recovery of flap shape, color and texture, significant differences with the original skin, or minor complications such as infection, but no effect on the outcome. Poor: TAM < 1.5, AOFSA ≤ 65, poor recovery of flap shape, color and texture, significant difference with the original skin, or complications such as serious infection, which have an impact on the efficacy. Overall effective rate = significant rate + general rate.

### 2.4. Statistical Analysis

Statistical Product and Service Solutions (SPSS) 23.0 (IBM, Armonk, NY, USA) was applied for statistical analysis. An independent sample *t*-test was used for comparison between groups for measurement data obeying normal distribution, and an independent sample *t*-test was used for comparison within groups, all expressed as ($\bar{x}$ ± *s*). Count data were tested by *χ*^2^ and expressed as rate (%). *P* < 0.05 indicates a statistical difference.

## 3. Results

### 3.1. Functional Recovery between the Two Groups

The preoperative TAM, AOFSA, and LEFS scores in the observation group were similar to those in the control group, and the difference was not statistically significant (*P* > 0.05). The postoperative TAM, AOFSA, and LEFS scores of the observers were higher than those of the control group, and the differences were statistically significant (*P* < 0.05) (Table 2).

### 3.2. Complications between the Two Groups

The number of patients with infection, skin graft necrosis, and subcutaneous hematoma in the observation group (total incidence rate 6.25%) was less (lower) than that in the control group (50.00%), and the differences had statistical significance (*P* < 0.05) (Table 3).

### 3.3. Clinical Efficacy of the Two Groups

The total number of patients with significant and general clinical efficacy (overall response rate 100.00%) in the observation group was more (higher) than that in the control group (68.75%), and the difference had statistical significance (*P* < 0.05) (Table 4).

## 4. Discussion

Skin with tendon defects in the hands, feet, and ankles are mostly caused by violent factors, such as scratches and car accidents due to falls from height [8,9]. The tendons are mostly located deep in the skin and involve many areas of severe skin lesions with bone and flesh visible. At the same time, tendons act as connective fibrous cords at the ends of muscles, by which muscles attach to bones or other structures and are important for maintaining motor function in the extremities [10]. And, the tendon was rich in blood supply, timely recovery of tendon defects, promoted the recovery of skin lesions, and motor function have a positive impact.

Conventional skin graft repair therapy promotes the restoration of traumatic skin color, elasticity, and texture by grafting full-thickness skin grafts on the autologous surface, with the advantages of less scarring and good cosmetic results. However, in practice, the risk of complications such as subcutaneous thrombosis, skin graft necrosis, and infection after conventional skin graft repair is generally high, and the results are limited in terms of tendon repair, which is not conducive to the recovery of motor function. Repair and treatment of lateral femoral circumflex vascular chimeric fascia lata flap: through transplantation of autologous fascia lata anterolateral thigh flap, it can effectively repair the tendon and soft tissue defects and can provide a good way for the transplanted flap, which plays an important role in promoting wound recovery [11].

In this study, the postoperative TAM, AOFSA, and LEFS scores of the observers were higher than those of the control group, suggesting that the repair of lateral femoral circumflex vessel chimeric fasciocutaneous flap can achieve better functional recovery. The reasons may be as follows: (1) Compared with conventional flap transplantation, the main trunk of the lateral thigh perforating vessels is more fixed, and the diameter is thick, the diameter of the harvested and transplanted vessels is about 4 cm, the survival rate is high and the anatomical structure is clear, the variation is less, the donor site is more concealed, and after harvesting the flap, it is not easy to cause excessive effects on the appearance and appearance of the patient [12]. (2) The characteristics of autologous fascia lata and tendon tissue are similar, and suturing the fascia lata and tendon at the defect site facilitates the recovery of tendon function [13]. And, fascia lata flap is conducive to isolating the skin and tendon after transplantation, can effectively reconstruct the deep tissue of the tendon, further reduce the degree of skin adhesion to the tendon, and is important to promote the recovery of function. Then, the suture is used to connect and suture the flap to carry the blood vessels, cutaneous nerves, and blood vessels and nerves at the defect site. Before vascular anastomosis, the flap carrying the blood vessels can provide a good barrier for the fascia lata. After vascular and nerve anastomosis, it can promote the recovery of blood supply and neurological function, facilitate the reconstruction of skin sensation in the recipient site, and further improve the recovery of postoperative motor function [14].

In terms of complications and therapeutic effect, this study showed that the total incidence rate of complications in the observation group was lower than that in the control group, and the total effective rate was higher than that in the control group, suggesting that the repair treatment of lateral thigh vascular chimeric fascia lata flap can reduce the risk of complications and improve the surgical efficacy. This may be because the flap carrying blood vessels can provide a better way for the transplanted flap, which is conducive to enhancing anti-infection and healing ability, and can effectively reduce the risk of complications such as infection and skin graft necrosis. Secondly, the skin color, texture, and elasticity of the foot and ankle of the same hand at the lateral femoral circumflex vessel are similar, which is conducive to the recovery of the color, texture, and elasticity of the skin tissue at the wound after transplantation, which can help the patient recover a better appearance and facilitate the improvement of cosmetic results. Yang et al. [15] studied that patients who received vascularized free anterolateral thigh fascia lata flap repair had better postoperative functional recovery and could recover more normal skin color and texture, which was consistent with the results of this study. It shows that the treatment of lateral femoral circumflex vessel chimeric fascia lata flap can achieve a significant surgical effect in the treatment of limb trauma, which is conducive to the recovery of function.

## 5. Conclusions

The application of lateral circumflex femoral artery embedded with fascia lata flap in the clinical diagnosis and treatment of hand, foot, and ankle skin with tendon defect can achieve ideal surgical efficacy. It can promote the recovery of hand tendon, ankle, and lower limb function, reduce the risk of complications, and improve the curative effect of surgery, which is worthy of popularization and application.

## Figures and Tables

**Table 1:** Comparison of basic data between the two groups (*x̅* ± *s*, *n*).

Group	*N*	Age (years)		Lesion area (cm^2^)		Tendon defect length (cm)		Gender composition	
		Scope	Average	Scope	Average	Scope	Average	Male	Female
Observation group	16	20–65	42.53 ± 7.76	30–128	79.09 ± 7.06	2–12	7.05 ± 1.04	10 (62.50%)	6 (37.50%)
Control group	16	18–61	39.57 ± 3.65	28–132	80.04 ± 8.12	2–11	6.59 ± 0.78	9 (56.25%)	7 (43.75%)
Χ^2^/*t*	—	1.381		0.353		1.415		0.130	
*P*	—	0.178		0.726		0.167		0.719	

**Table 2:** Comparison of functional recovery of the two groups (*x̅* ± *s*, points).

Group	*N*	TAM		AOFSA		LEFS	
		Preop	Postop	Preop	Postop	Preop	Postop
Observation group	16	0.98 ± 0.23	2.46 ± 0.31	48.83 ± 5.34	76.43 ± 6.89	43.64 ± 5.46	71.24 ± 6.75
Control group	16	0.95 ± 0.18	1.62 ± 0.28	49.03 ± 5.83	66.82 ± 5.97	44.01 ± 6.04	62.11 ± 6.43
*T*	—	0.411	8.043	0.101	4.217	0.182	3.917
*P*	—	0.684	0.001	0.920	0.001	0.857	0.001

**Table 3:** Comparison of complications between the two groups [*n*, (%)].

Group	Number of subjects	Infection	Skin graft necrosis	Subcutaneous hematoma	Total occurrence
Observation group	16	1 (6.25%)	0	0	1 (6.25%)
Control group	16	4 (25.00%)	2 (12.50%)	2 (12.50%)	8 (50.00%)
Χ^2^	—	2.133	2.133	2.133	7.930
*P*	—	0.144	0.144	0.144	0.047

**Table 4:** Clinical efficacy comparison between the two groups (*n*, (%)).

Group	*N*	Significant	General	Poor	Overall response rate
Observation group	16	9 (56.25%)	7 (43.75%)	0	16 (100.00%)
Control group	16	2 (12.50%)	9 (56.25%)	5 (31.25%)	11 (68.75%)
Χ^2^	—	6.788	0.500	5.926	9.705
*P*	—	0.009	0.480	0.015	1.8

## Data Availability

The datasets used and analyzed during the current study are available from the corresponding author on reasonable request.
